The article "HGF/c-Met Promote Renal Carcinoma Cancer Stem Cells Enrichment Through Upregulation of Cir-CCDC66" was published in 2020. Journal: Technol Cancer Res Treat.

# HGF/c-Met Promote Renal Carcinoma Cancer Stem Cells Enrichment Through Upregulation of Cir-CCDC66

**DOI:** 10.1177/1533033819901114

**Published:** 2020-01-29

**Authors:** Juhong Yang, Lei Yang, Shen Li, Ning Hu

**Affiliations:** 1 Department of Nephrology, The First People’s Hospital of Jingmen, Jingmen, Hubei, China; 2 Department of Urology Surgery, The First People’s Hospital of Jingmen, Jingmen, Hubei, China; 3 Department of Cardiovascular, The First People’s Hospital of Jingmen, Jingmen, Hubei, China

**Keywords:** HGF/c-Met, cir-CCDC66, cancer stem cell, renal carcinoma cancer

## Abstract

Increasing studies have suggested that circular RNAs play an important function in the process of numerous cancers. We aimed to investigate the possible role of cir-CCDC66 in renal carcinoma cancer. As cancer stem cells are responsible for the renal carcinoma cancer tumor growth and resistance to conventional therapy, we focus on the cir-CCDC66 influence on renal carcinoma cancer stem cells. In this study, we performed experiments in human renal tubular epithelial cell HK2 cells and several renal carcinoma cancer cancer cell lines. The results showed that cir-CCDC66 was upregulated not only in renal carcinoma cancer cancer cell lines but also in cancer stem cell spheres. What’s more, the results showed that cir-CCDC66 enhanced the cancer stem cell enrichment. Further mechanistic studies showed that hepatocyte growth factor/c-Met pathway was activated in cancer stem cell enrichment and responsible for the cir-CCDC66 upregulation. Inhibition of hepatocyte growth factor/c-Met could block cir-CCDC66-induced cancer stem cell enrichment. In conclusion, our research revealed a novel mechanism between hepatocyte growth factor/c-Met/cir-CCDC66 and cancer stem cell enrichment. We verified that cir-CCDC66 could be a promising biomarker and therapy target for renal carcinoma cancer treatment.

## Introduction

Renal cell carcinoma (RCC) accounts for almost 90% of kidney tumors and 2% to 3% of all malignant cancers worldwide.^1^ The incidence of RCC is increasing at a rate of about 2% year by year. The standard treatment of RCC is mainly surgery. The prognosis of RCC is very poor as the 5-year survival rate is only about 5% despite the surgical resection. Additionally, almost 40% of patients with RCC developed recurrence after the surgery.

Renal carcinoma cancer is not an entity, it comprises different populations of tumors that originate from the highly heterogeneous epithelium of renal tubules. The mechanisms of metastasis and recurrence remain unclear.^2^ Cancer stem cell (CSC) theory may be one of the possible mechanism.

Cancer stem cells are the small population with multipotential capacity such as self-renew ability and high tumorigenic activity. What’s more, CSCs play important roles in the chemoresistance and recurrence, which are the main causes of high mortality. Cancer stem cell–targeted therapy may bring new hope for patients with RCC.

The article "HGF/c-Met Promote Renal Carcinoma Cancer Stem Cells Enrichment Through Upregulation of Cir-CCDC66" was published in 2020. Journal: Technol Cancer Res Treat.

Circular RNAs (cirRNAs) are now found as a novel kind of noncoding RNAs with the development of next-generation sequencing and bioinformatics technology. The cirRNAs are widely expressed in numerous cancers with diverse functions. The cirRNAs are closed loops, which help stabilize the RNA to be resistant to RNase digestion. The cirRNA can bind to microRNAs as miRNA sponge to block the digestion of targeted genes. Therefore, because of structure stability, tissue-specific expression, and high abundance, cirRNA could function as biomarkers or therapy targets for cancers.

We selected several circular RNA for the cancer investigation because of their important role in cancer. The presence of selected RNAs was identified by reverse transcription polymerase chain reaction (RT-PCR) in 8 renal carcinoma cells and 1 normal kidney cell line. We chose cir-CCDC66, which was expressed in all cells, as our research object. Cir-CCDC66 (ID, hsa_circ_0001313) has 468 nucleotides and is located in chr3:56626997-56628056. At present, it is widely known that pre-mRNA could be transcribed into linear noncoding RNAs, but pre-mRNA also can be nonlinearly spliced into circRNA. CircCCDC66 is nonlinearly spliced from the CCDC66 pre-mRNA. It has been reported that the expression of circCCDC66 does not affect the level of the linear transcript in either overexpression or specific knockdown of circCCDC66.^3^ It also has been reported that the expression of linear CCDC66 in tumor specimens is not correlated with circCCDC66 in colon cancer. It has been showed that circ-CCDC66 is overexpressed in several cancers such as colon cancer and lung adenocarcinoma.^3,4^ The studies demonstrate that the upregulation of circ-CCDC66 is closely related to poor prognosis and accelerates the malignant process of cancer. As the reports of the function of circ-CCDC66 are very limited. In our work, we explored the function of circ-CCDC66 in RCC and the possible mechanism.

## Materials

### Cell Culture

Renal cancer cell lines Caki-1, Caki-2,786-O, 767P, and normal human renal tubular epithelial cell HK2 were obtained from The Global Bioresource Center cell bank. OS-RC-2, SN12C, SKRC39, ACHN, and A498 were purchased from Type Culture Collection of Chinese Academy of Sciences. The basic culture medium for 786-O, 769P, and SKRC39 OS-RC-2 was RPMI-1640 (Gibco, Grand Island, NY). The basic culture medium for Caki-1 and ACHN was Dulbecco’s Modified Eagle Medium (DMEM; Gibco). The basic culture medium for Caki-2 was McCoy’s 5A. All the cancer cell lines were cultured in basic medium with 10% fetal bovine serum. HK2 was cultured by Invitrogen kit (Catalog Number 17005-042).

The article "HGF/c-Met Promote Renal Carcinoma Cancer Stem Cells Enrichment Through Upregulation of Cir-CCDC66" was published in 2020. Journal: Technol Cancer Res Treat.

### Cell Proliferation Assay

We inoculated 3000 renal cancer cells into each well of a 96-well plate. After the cells attached to the plates, we added 10 μL of cell counting kit 8 (CCK8) per well. After 3 hours, the optical density value at 450 nm was measured.

### Sphere-Forming Assay

The cancer cells were prepared for single cells. The sphere-forming medium was cultured in DMEM/F12 medium contained 0.4% bovine serum albumin (Sigma [Sigma-Aldrich, St. Louis, MO, USA]), supplemented with 25 ng/mL epithelial growth factor, 25 ng/mL basic fibroblast growth factor-2, and 50 μg/mL insulin and 1 × B27. One thousand single cells were plated per well in 24-well plates with ultralow attachment. The cell spheres were counted and taken photos of 10 days later.

### Drugs

SU11274, hepatocyte growth factor (HGF; Sigma) were dissolved and stored according to the instruction.

### Antibody

c-Met antibody was obtained from Invitrogen and Phospho-Met (Tyr1349) antibody was from Cell Signaling Technology.

### Silencing of Gene Expression

Silence of cirRNA CCDC66 (cirRNA CCDC66 KD) was carried out by direct delivery of small interfering RNA (siRNAs; si-cir-CCDC66 and si-cir-CCDC66) in RCC cancer cells. The overexpression of cir-CCDC66 was carried out with transfection of cir-CCDC66 plasmids. The siRNAs and cir-CCDC66 plasmids all from Genewiz Company (Suzhou, China). All the transfections were carried out with Lippo3000 Kit (Thermo Fisher Scientific).

### RNA Extraction and Quantitative Reverse Transcription Polymerase Chain Reaction

Total RNA of renal cancer cells were extracted by Trizol Kit of Invitrogen. The Total RNA (10 μg) was incubated with 40U RNase R (Epicenter Technologies, Madison, Wisconsin) at 37°C for 1 hour. After treatment with RNase R, the product of RNA was determined by quantitative reverse transcription–polymerase chain reaction (qRT-PCR). Quantitative reverse transcription polymerase chain reaction were then carried out with Power SYBR Green PCR Master mix kit of Roche (Roche Applied Science, Basel, Switzerland), according to the manuscript instructions. 2^−ΔΔCt^ method was used to analyze the RNA levels. The PCR conditions are as follows: 95°C, 5 minutes; 95°C, 15 seconds, 40 cycles; 53°C, 30 seconds; 72°C, 35 seconds. The primers are as followings^5,6^:

**Table:** 

Gene	Forward (5′-3′)	Reverse (5′-3′)
Circ-CCDC66	TCTCTTGGACCCAGC TCA	TGAATCAAAGTGCA TTGCCC
CCDC66	AAATGAGCATGCCAT TTCT	CTTGGCTAAAAATA AATCTG
GAPDH	AGCCACATCGCTCAG ACA	GCCCAATACGACCA AATCC

The article "HGF/c-Met Promote Renal Carcinoma Cancer Stem Cells Enrichment Through Upregulation of Cir-CCDC66" was published in 2020. Journal: Technol Cancer Res Treat.

### Western Blot

The protein levels were identified by Western blot. The lysis buffers were prepared: 15 mM ethylenediaminetetraacetic acid, 120 mM NaCl, 0.1 mM sodium orthovanadate, 25 mM 3-(N- morpholine) sodium propionate salt (MPOS), 0.1% Triton X-100, 15 mM MgCl_2_, and 1% protease inhibitor cocktail. The lysates of cells were separated by sodium dodecyl sulfate-polyacrylamide gel electrophoresis, then the protein was transferred to the negative control (NC) membrane.

### Statistical Analysis

All statistical analyses were carried out using GraphPad Prism 5 software. Each result is shown as the mean ± standard deviation (n = 3). The statistical significance of comparisons among multiple groups was assessed by 1-way analysis of variance, followed by least-significant difference *t* test analysis, with *P* < .05 considered to be statistically significant (*.05, **<.01, and ***<.001).

## Results

### Identification of Cir-CCDC66 in Renal Carcinoma

As there were no previous reports on the expression of cir-CCDC66 in renal carcinoma, we carried out the qRT-PCR to identify the presence of cir-CCDC66 in renal carcinoma. In order to confirm the PCR amplification products were circular RNAs not linear RNAs, we applied RNase R enzyme that only digests linear RNAs but not circular RNAs to treat the RNA before PCR experiments.^7^ The results showed that circular CCDC66 had higher resistance to the RNase R enzyme compared to the linear CCDC66 (Figure 1A). Further, we identified the expression level of circ-CCDC66 in several RCC cell lines. The results showed that cir-CCDC66 was upregulated in renal carcinoma cells than the normal kidney cells (Figure 1B).

**Figure 1.** Identification of cir-CCDC66 in RCC cancer cell lines. A, qRT-PCR was carried out toidentify linear CCDC66 and circular CCDC66 expression in the RCC cancer cell line 767P. B, qRT-PCR was carried out to identify the expression of cir-CCDC66 in different RCC cell lines. Data are shown as the mean (SD; n = 3). qRT-PCR indicates quantitative reverse transcription polymerase chain reaction; RCC, renal carcinoma cancer; SD, standard deviation.

### Cir-CCDC66 Is Enriched in CSC Spheres

To assess the role of circular CCDC66 in RCC CSCs, we used cell sphere assay to enrich the CSCs. Sphere-forming assay has been reported as one of the important methods for RCC CSCs identification. The RCC cells were plated in cell sphere conditional culture medium in 24-well plates at a density of 1000 cells/well. With the cell sphere conditional medium and nonadherent culture dish, the CSCs grew as 3-dimensional spheres. We carried out qRT-PCR to identify the expression of circular CCDC66 in RCC parental and CSCs at day 0, day 4, and day 8. The results showed that circular CCDC66 RNA was upregulated in CSCs than the parental cells. What’s more, circular CCDC66 expression increased with time (Figure 2A and B).

The article "HGF/c-Met Promote Renal Carcinoma Cancer Stem Cells Enrichment Through Upregulation of Cir-CCDC66" was published in 2020. Journal: Technol Cancer Res Treat.

**Figure 2.** cir-CCDC6 is upregulated in the cancer stem cells. We inoculated cancer cells in normal medium and cancer stem cell culture medium and detected mRNA levels of cir-CCDC66 in different days by qRT-PCR. A, The mRNA level of cir-CCDC66 in 767P. B, The mRNA level of cir-CCDC66 in Caki-1. Data are shown as the mean ± SD (n = 3). qRT-PCR indicates quantitative reverse transcription polymerase chain reaction; SD, standard deviation.

### Renal Carcinoma CSCs Enrichment Dependent on Cir-CCDC66

To figure out the function of cir-CCDC66 in CSCs enrichment, we knocked out cir-CCDC66 with transfection of cir-CCDC66 siRNAs and overexpressed cir-CCDC66 with transfection of plasmids in RCC cancer cell lines. Real-time PCRs were carried out to identify the expression of cir-CCDC66 in RCC cell lines (Figure 3A, D, G, and J). CCK8 assay results showed that silence of cir-CCDCC66 leaded to the inhibition of tumor cells growth (Figure 3B and E). To assess the influence of cir-CCDC66 on CSC frequency, we carried out CSC assays. Notably, cir-CCDC66 silence was associated with an obvious reduction in the CSC sphere numbers in 767P (Figure 3C) and SKRC390 ACHN (Figure 3F).

To further validate the contribution of cir-CCDC66 in CSC enrichment, we overexpressed cir-CCDC66 in Caki-1 (Figure 3G) and OS-RC-2(Figure 3J). The overexpression of cir-CCDC66 promoted the cell growth of Caki-1 (Figure 3H) and OS-RC-2(Figure 3K).What is more, cir-CCDC66 enhanced the CSC frequency (Figure 3I and L). Totally, our experiments validated that cir-CCDC66 could promote the RCC cancer cell growth rate and enhance CSC frequency. c-Met was activated in CSC enrichment. Previous experiments have shown that cir-CCDC66 plays an important role in the enrichment and frequency of RCC CSCs. The results showed that cir-CCDC66 was upregulated in cancer cells. Most of the recent research studies focus on the downstream of cir-CCDC66; we want to know the mechanism of cir-CCDC66 upregulation. As the research reported that cirRNA CCDC66 was positively regulated by c-Met in lung adenocarcinoma cells.

**Figure 3.** cir-CCDC66 contributes to the RCC cancer stem cell enrichment. A-F, Transfection of NC-siRNA or circ-CCDC66-siRNA was carried out in 767P (A) and SKRC39 (D) RCC cancer cell lines. Transfection efficacy of circ-CCDC66-siRNA and NC-siRNA in 767P (A) and SKRC39 (D) were detected by qRT-PCR. CCK8 was used to detect the growth in 767P (B) and SKRC39 (E). Cell sphere assays were carried out in 767P(C) and SKRC39 (F). G-L, Transfection of vector or circ-CCDC66 was carried out in Caki-1and OS-RC-2 RCC cancer cell lines. Transfection efficacy was detected by RT-PCR in Caki-1(G) and OS-RC-2(J) RCC cancer cell lines. CCK8 was used to detect the growth in Caki-1(H) and OS-RC-2(K). Cell sphere assays were carried out in Caki-1(I) and OS-RC-2(L). qRT-PCR indicates quantitative reverse transcription polymerase chain reaction; RCC, renal carcinoma cancer; siRNA, small interfering RNA; CCK8, cell counting kit 8; NC, negative control;

The article "HGF/c-Met Promote Renal Carcinoma Cancer Stem Cells Enrichment Through Upregulation of Cir-CCDC66" was published in 2020. Journal: Technol Cancer Res Treat.

### C-Met Is Activated in RCC CSC Enrichment

Mesenchymal–epithelial transition factor c-Met is the receptor for HGF receptor. c-Met is a transmembrane tyrosine kinase. c-Met and its ligand HGF could bind together to form a homodimer that can cause tyrosine phosphorylation accompanied with multiple downstream signaling pathways activation. c-Met plays important roles in regulation of cell growth, survival, and metastasis.^8^ Abnormal activation of c-Met signaling pathway was detected in many malignant tumors, including gastric cancer, lung cancer, esophageal cancer, breast cancer, liver cancer, colon cancer, prostate cancer, pancreatic cancer, kidney cancer, ovarian cancer, glioma, melanoma, osteosarcoma, and various cancers. Recent studies have found that c-Met activation is in close relationship with the occurrence and development of malignant tumors.^9-11^ What’s more, c-Met has been reported to be a new biomarker for pancreatic CSCs.^12^ It has been reported HGF/c-Met could promote epithelial-to-mesenchymal transition (EMT) in lung adenocarcinoma cells through cirCCDC66 indicating the important role of HGF/c-Met/circ-CCDC66 in cancers.^4^ What’s more, c-Met has been reported to promote bone metastasis development induced by renal CSCs and enhance the CSCs factors expression in colon cancers.^13-15^

To confirm the relationship between c-Met and CSCs, we carried out Western blot to identify the c-Met activation in RCC CSC enrichment. The results showed that the c-Met phosphorylation was upregulated with increasing time in the CSC culture compared to common medium in 767P (Figure 4A) and SKRC39 ACHN (Figure 4B). The results indicate that c-Met activation plays important roles in RCC CSC formation.

**Figure 4.** c-Met is activated in cancer stem cell formation. A, 767P was cultured in common medium and cancer stem cell medium for indicated days. Western blot was carried out to detect phosphorylation and total level of c-Met. B, Caki-1 was cultured in common medium and cancer stem cell medium for indicated days. Western blot was carried out to detect phosphorylation and total level of c-Met.

The article "HGF/c-Met Promote Renal Carcinoma Cancer Stem Cells Enrichment Through Upregulation of Cir-CCDC66" was published in 2020. Journal: Technol Cancer Res Treat.

### C-Met Promotes the Cir-CCDC66 Expression and CSC Enrichment

As the results showed that c-Met expression was enhanced in the CSC formation process, the role of HGF/c-Met pathway in cir-CCDC66-induced CSCs enrichment remained unclear. In 767P cells, we silenced the expression of c-Met by siRNA transfection. Western blot was used to identify the expression of total and phosphorylation of c-Met (Figure 5A). Then, we detected the mRNA of cir-CCDC66 by qRT-PCR. The results showed that silence of c-Met leaded to the reduction in cir-CCDC66 mRNA level (Figure 5B) accompanied with decreased CSC number (Figure 5C). Then, we added HGF to activate the HGF/c-Met pathway and the results showed that HGF could promote the mRNA level of cir-CCDC66 and CSC numbers in 767P NC cells, whereas HGF could not influence the cir-CCDC66 and CSC numbers in 767 si-c-Met cells. The results showed that c-Met and cir-CCDC66 contribute to the RCC CSC together. To confirm the function of HGF/c-Met/cir-CCDC66, we overexpressed c-Met in Caki-1 and then inhibited the phosphorylation of c-Met by SU11274 (Figure 5D). The data showed that the overexpression of c-Met could significantly increase the cir-CCDC66 mRNA level and CSCs number (Figure 5E and F). What’s more, inhibition of c-Met activation could block the increase of cir-CCDC66 and CSC sphere formation. All the results above came to a conclusion that c-Met could influence the cir-CCDC66 expression and CSC.

**Figure 5.** c-Met promotes the expression of cir-CCDC66 and cancer stem cell enrichment. A, c-Met was silenced in 767P (left) and then the c-Met was activated by 10 ng/mL HGF (right). Western blot was used to identify the activation of c-Met. B, RT-PCR was used to identify the expression level of cir-CCDC66. C, Cell sphere assays were carried out to detect the cancer stem cell frequency. D, c-Met was overexpressed in Caki-1 cells (left) and then treated with 10 nM c-Met inhibitor SU11274 (right). Western blot was used to identify the transfection and inhibition efficacy. E, RT-PCR was used to identify the expression level of circ-CCDC66 in Caki-1. F, Cell sphere assays were carried out to detect the cancer stem cell frequency in Caki-1. HGF indicates hepatocyte growth factor; RT-PCR, quantitative reverse transcription polymerase chain reaction.

### C-Met Induces CSCs Enrichment Dependent on Cir-CCDC66

To confirm the function of cir-CCDC66 in c-Met-induced CSC enrichment, we carried out the rescue experiments in 767P and Caki-1 RCC cells. As the data showed, reexpression of cir-CCDC66 in 767P-si-c-Met cells could totally rescue the CSC enrichment (Figure 6A). In Caki-1, silence of cir-CCDC66 could block the CSC enrichment induced by c-Met overexpression (Figure 6B). The rescue experiments verified that c-Met promoted the CSC enrichment through cir-CCDC66. All data above showed that c-Met/cir-CCDC66 pathway was critically important in RCC CSCs enrichment.

The article "HGF/c-Met Promote Renal Carcinoma Cancer Stem Cells Enrichment Through Upregulation of Cir-CCDC66" was published in 2020. Journal: Technol Cancer Res Treat.

**Figure 6.** c-Met induces cancer stem cells enrichment dependent on cir-CCDC66. A, Cir-CCDC66 or vector was transfected in 767P-si-c-Met cells. Cell sphere assays were carried out in 767P cells. B, si-circ-CCDC66 or NC-siRNAs was transfected in Caki-1-OE-c-MET cells. Cell sphere assays were carried out in Caki-1 cells. siRNA indicates small interfering RNA.

## Discussion

CircRNAs are a newly found group of noncoding RNAs with covalently closed loop structures. The biological functions of circRNA were largely unknown.^16^ Highly conserved sequences and resistance to RNase are the important properties. The circRNA could exist over 48 hours, which is much longer than the mRNA. The stability of structure allows the circRNA to play important roles in cell activities. Now, increasing reports demonstrate that circRNAs act as important players in complicated physiological and pathological processes in various cancers.^17^

It has been reported that cir-CCDC66 plays important roles in colon cancer proliferation and migration.^3^ Circular RNA CCDC66 promote cancer growth, metastasis, and EMT in lung cancer.^4^ However, no research has focus on the function of cir-CCDC66 in RCC.

In our research, we detected the expression of cir-CCDC66 in several RCC cancer cell lines and found that cir-CCDC66 was with higher expression level in RCC cancers cell lines than normal renal cells (Figure 1). What’s more, the results showed that the RCC CSC spheres had high level of cir-CCDC66 expression than the RCC cancer cells suggesting that cir-CCDC66 was upregulated in CSCs (Figure 2). Further study showed that overexpression of cir-CCDC66 could promote the cell growth and increase RCC CSC frequency while silence of cir-CCDC66 reduce cell growth rate and CSC numbers (Figure 6). All these data together showed cir-CCDC66 could promote CSC enrichment.

Cancer stem cell research studies are expanding rapidly because of important function in various cancer types. Currently, increasing data demonstrate cell sphere culture to be an important method to enrich CSCs because of its property of anchorage-independent growth. Various CSC subpopulations have been enriched by application of cell sphere culture.^18,19^ No research has reported about the relationship between cir-CCDC66 and CSCs. We found that cir-CCDC66 promoted CSC in RCC cancer. Cir-CCDC66 may be a promising target for cancer therapy.

As the cir-CCDC66 is highly expressed in RCC cancer cells, we want to know the mechanism of abnormal expression of cir-CCDC66. The reports showed that cir-CCDC66 expression was positively regulated by HGF/c-Met in lung adenocarcinoma cells.^4^ Whether HGF/c-Met could regulate cir-CCDC66 expression in RCC remained unclear.

The article "HGF/c-Met Promote Renal Carcinoma Cancer Stem Cells Enrichment Through Upregulation of Cir-CCDC66" was published in 2020. Journal: Technol Cancer Res Treat.

In our research, we found that c-Met pathway was upregulated in CSC enrichment. Silence of c-Met blocked the cir-CCDC66 expression and CSC frequency and overexpressed c-Met increased cir-CCDC66 expression and CSC frequency (Figure 4). What’s more, reexpressed the cir-CCDC66 in si-c-Met cells could rescue the CSC number (Figure 5A). Silence of cir-CCDC66 could block the c-Met-induced CSC enrichment (Figure 5B). These data verified the important role of c-Met/cir-CCDC66 in RCC CSC enrichment. c-Met has been a prognostic marker and potential therapeutic target in RCC.^20^ We provided a new mechanism for HGF/c-Met-induced CSCs. Our researcher suggested that the combination of c-Met inhibitor and cir-CCDC66 inhibitor may be a new therapy for RCC.

As a novel star, circRNAs play important roles in numerous cancers. Our research have investigated the mechanism of a new pathway in regulation of RCC CSCs. Our research showed that HGF/c-Met/cir-CCDC66 played important roles in RCC CSC enrichment that provided a new insight into CSC. Combination of c-Met inhibition and cir-CCDC66 would be a promising therapeutic target for RCC.

## Abbreviations

cirRNA: circular RNAs
CSC: cancer stem cell
DMEM: Dulbecco Modified Eagle Medium
EMT: epithelial-to-mesenchymal transition
HGF: hepatocyte growth factor
RCC: renal carcinoma cancer

## References

[1] DolgushinMKornienkoVProninI Renal Cell Carcinoma (RCC). Cham, Switzerland: Springer; 2018.

[2] YuanZXMoJZhaoGShuGFuHLZhaoW Targeting strategies for renal cell carcinoma: from renal cancer cells to renal cancer stem cells. Front Pharmacol. 2016;7:423.2789109310.3389/fphar.2016.00423PMC5103413

[3] MemczakSJensMElefsiniotiA, et al. Circular RNAs are a large class of animal RNAs with regulatory potency. Nature. 2013;495(7441):333–338.2344634810.1038/nature11928

[4] JosephNAShiow-HerCZoeL, et al. The role of HGF-MET pathway and CCDC66 cirRNA expression in EGFR resistance and epithelial-to-mesenchymal transition of lung adenocarcinoma cells. J Hematol Oncol. 2018;11(1):74.2985533610.1186/s13045-018-0557-9PMC5984410

[5] HsiaoKYLinYCGuptaSK, et al. Noncoding effects of circular RNA CCDC66 promote colon cancer growth and metastasis. Cancer Res. 2017;77(9):2339–2350.2824990310.1158/0008-5472.CAN-16-1883PMC5910173

[6] DekomienGVollrathCPetrasch-ParwezE, et al. Progressive retinal atrophy in Schapendoes dogs: mutation of the newly identified CCDC66 gene. Neurogenetics. 2010;11(2):163–174.1977727310.1007/s10048-009-0223-z

The article "HGF/c-Met Promote Renal Carcinoma Cancer Stem Cells Enrichment Through Upregulation of Cir-CCDC66" was published in 2020. Journal: Technol Cancer Res Treat.

[7] HossainSTMalhotraADeutscherMP How RNase R degrades structured RNA. J Biol Chem. 2016;291(15):7877–7887.2687296910.1074/jbc.M116.717991PMC4824996

[8] BirchmeierCBirchmeierWGherardiEVande WoudeGF Met, metastasis, motility and more. Nat Rev Mol Cell Biol. 2003;4(12):915–925.1468517010.1038/nrm1261

[9] LiJFNiuYXingYLiuF A novel bispecific c-MET/CTLA-4 antibody targeting lung cancer stem cell-like cells with therapeutic potential in human non-small cell lung cancer. Biosci Rep. 2019;39(5): BSR20171278.2918758410.1042/BSR20171278PMC6542762

[10] JunHJBronsonRTCharestA Inhibition of EGFR induces a c-MET-driven stem cell population in glioblastoma. Stem Cells. 2014;32(2):338–348.2411521810.1002/stem.1554PMC4442493

[11] YashiroMNishiiTHasegawaT, et al. A c-Met inhibitor increases the chemosensitivity of cancer stem cells to the irinotecan in gastric carcinoma. Br J Cancer. 2013;109(10):2619–2628.2412923510.1038/bjc.2013.638PMC3833223

[12] LiCHynesMDoschJWuJJSimeoneDM Abstract LB-257: c-Met: a new cancer stem cell marker and therapeutic target for pancreatic cancer. Cancer Res. 2011;70:257.

[13] LiCWuJHynesM, et al. C-met is a marker of pancreatic cancer stem cells and therapeutic target. Gastroenterology. 2011;141(6):2218–2227.e5. 2186447510.1053/j.gastro.2011.08.009

[14] D’AmicoLBelisarioDMigliardiGGrangeCRoatoI C-met inhibition blocks bone metastasis development induced by renal cancer stem cells. Oncotarget. 2016;7(29):45525–45537.2732255310.18632/oncotarget.9997PMC5216739

[15] ChatziioannouMApostolouPToloudiM, et al. 310 Comparative study of Nanog, Oct3/4 and sox2 gene expression following C-met gene knockdown in colon cancer stem cells. Eur J Can. 2012;48(6):95.

[16] ChenLLYangL Regulation of circRNA biogenesis. RNA Biol. 2015;12(4):381–388.2574683410.1080/15476286.2015.1020271PMC4615371

[17] Gla ArPPapavasileiouPRajewskyN Circbase: a database for circular RNAs. RNA. 2014;20(11):1666–1670.2523492710.1261/rna.043687.113PMC4201819

[18] ZhangSBalchCChanMW, et al. Identification and characterization of ovarian cancer-initiating cells from primary human tumors. Cancer Res. 2008;68(11):4311–4320.1851969110.1158/0008-5472.CAN-08-0364PMC2553722

[19] RappaGMercapideJAnzanelloF, et al. Growth of cancer cell lines under stem cell-like conditions has the potential to unveil therapeutic targets. Exp Cell Res. 2008;314(10):2110–2122.1842360510.1016/j.yexcr.2008.03.008PMC2677207

[20] GibneyGTAzizSACampRL, et al. C-Met is a prognostic marker and potential therapeutic target in clear cell renal cell carcinoma. Ann Oncol. 2013;24(2):343–349.2302299510.1093/annonc/mds463PMC3551486

